# Evaluation of *Pleurotus* Mushroom Effects on Histopathological Changes in Organs of Diabetic Rats

**DOI:** 10.1155/2023/1520132

**Published:** 2023-04-14

**Authors:** Sushil Kumar Dubey, Sachchida Nand Rai, Vinay Kumar Singh, Anand Kumar Bajpeyee, M. P. Singh

**Affiliations:** ^1^Centre of Biotechnology, University of Allahabad, Prayagraj 211002, India; ^2^Department of Zoology, C.M.P. Degree College, University of Allahabad, Prayagraj 211002, India

## Abstract

Diabetes mellitus (DM) is a metabolic disorder that can be categorized mainly into type 1 and type 2. Diabetes type 1 is caused due to *β*-cell destruction, whereas type 2 is caused by the resistance of cell receptors. Many therapies are available for the management of diabetes, but they have some side effects, and as a result of this, people are attracted to natural treatments. *Pleurotus* mushrooms are well documented for their medicinal attributes and their role in the treatment of diseases like cancer, infectious disease, neurodiseases, and inflammatory disease. The protective mechanism of the *Pleurotus fossulatus* (*P. fossulatus*) mushroom and its detailed histological study on kidneys and the liver in diabetic conditions were unexplored. The present study evaluated the effects of *P. fossulatus* aqueous extract on histological changes in the diabetic rat model. Male Wistar albino rats were used to create the diabetic model by using streptozotocin (STZ) intraperitoneal (IP) injection. The animals were separated into five different groups, with six animals in each. Only group I, animals that did not receive STZ, was considered a normal control. Group II was a diabetic control and received normal saline, and group III was a drug control and received metformin as a standard drug. Groups IV and V were dosing groups, which received the aqueous extract of *P. fossulatus* in 250 mg/kg and 500 mg/kg of body weight concentrations, labeled as T1 and T2 groups, respectively. The T1 and T2 groups clearly showed their potential to reverse the histopathological changes in the kidney and liver. However, the T2 group was more effective than the T1 group, as results indicate that functions of the glomerulus and its structural deformity were restored to their near-natural form in the T2 group. In the case of the liver, the histological changes like the dilatation of sinusoids, more numbers of the Kupffer cell formation, and necrosis were restored in the T2 group. All these results proved the potential of *P. fossulatus* against the side effects of diabetes. It could protect the organs from developing diabetic nephropathy (DN) and liver-related diseases like cirrhosis and nonalcoholic fatty liver disease (NAFLD).

## 1. Introduction

Diabetes mellitus (DM) is defined as a metabolic disorder caused by less insulin secretion or impaired insulin action [1]. DM is generally categorized into type 1 and type 2. Diabetes type 1 is caused by the antibody-mediated self-destruction of *β*-cells. Hence, it is called autoimmune-mediated DM. On the other side, diabetes type 2 is developed due to the resistance of receptors, present in peripheral tissues, against insulin action [2]. Pancreatic *β*-cells are responsible for the secretion of insulin which helps to metabolize the glucose and prevents raising the level of glucose. Due to hyperglycemic conditions, several pathological complications cause retinopathy, cardiovascular diseases, cancer, neuropathy, nephropathy, renal dysfunction, and even can cause death if it is uncontrolled and untreated [3, 4]. In hyperglycemic conditions, the liver and kidney are the most affected organs in which many biochemical and histological changes can be observed.

DN is a condition in which the glomerular filtration rate (GFR) declined continuously, and it leads to end-stage renal disease (ESRD). This can also increase the risk of cardiovascular diseases and infection-related complications [5]. The histological changes related to diabetes nephropathy (DN) can be detected two years after diabetes is diagnosed, and both types of diabetes can cause DN. According to a study on the diabetic rat model, lipofuscin pigment excess expression is a sign of cell injury [6]. The subnuclear lipid vacuolization or glycogen deposition leads to a stressful condition that ultimately caused cell damage. In the severe condition of hyperglycemia, the accumulation of glycogen in tubule cells is called the Armanni-Ebstein cells [7]. During diabetes type 1, some histological changes can be observed in renal tubules, arterioles, mesangial expansion, interstitium, podocytes, and thickening of glomerular basement membrane (GBM). On the other side, in diabetes type 2, glomerulopathies with minimal lesion nephropathy, diabetic glomerulosclerosis, and mesangial proliferative glomerulonephritis can be observed from the initial to advanced stages [8].

Many researchers have revealed that DM can be linked to many liver-associated disorders like an abnormal accumulation of hepatic enzymes, cirrhosis, carcinomas, NAFLD, and acute liver disease. Moreover, the accumulation of excess fat in the liver called steatosis can worsen metabolic dysfunction. Microvesicular steatosis is a condition in which the fats displaced the cytoplasm of the liver and in advanced stages, and the fats distort the nucleus called macrovesicular steatosis. Some other histological changes can be seen as mild lymphocytic, abnormal numbers of the Kupffer cells, and neutrophils. Generally, about 3% of patients experience symptoms like fibrosis, hepatic inflammation, and necrosis; these conditions are defined as nonalcoholic steatohepatitis (NASH). All these conditions are collectively called steatohepatitis [9]. Some other degenerative histological changes can also be found as hepatocyte vacuolation, dilatation of sinusoidal spaces, and irregular size of nuclei [10].

There are many drugs including insulin present in the market which can be taken either through oral or by injection. These medicines have some side effects which have already been reported in many kinds of research. So, due to all these problems, people are searching for herbal and fewer side-effect-causing medicines. *Pleurotus* species are generally grown on decayed maters of trees and agricultural waste products in wild conditions and can be cultivated in lab conditions as well. This mushroom was discovered for the first time in India and is characterized as white-rot fungi. The species of these mushrooms have been consumed for centuries for their pleasant taste, entomopathogenic properties, and culinary effect. It contains many ethnopharmacological values as it has biomolecules like proteins, vitamin B complex (folic acid, thiamin, and riboflavin), minerals (Fe, Ca, P, and Se), and polysaccharides (*β*-glucan). Due to all these medicinal properties, *Pleurotus* mushrooms can show a good synergistic effect on the liver and kidney in diabetic conditions [11].

We have reported that the biochemical changes in the liver and kidney can be controlled by the aqueous extract of *Pleurotus fossulatus* (*P. fossulatus*) in our previous study [12]. The objective of this study was to determine the histopathological changes and protective effects of *P. fossulatus* aqueous extract from hyperglycemia on the liver and kidney in streptozotocin- (STZ-) induced diabetic rat modal.

## 2. Materials and Methods

### 2.1. *P. fossulatus* Aqueous Extract Preparation

The mushroom fruiting bodies were collected from the mushroom laboratory, Centre of Biotechnology, University of Allahabad, Prayagraj, India. The fruiting bodies were rinsed with potable tap water twice and sprayed in the shade until completely air-dried, and then, the fine powder was prepared by using a mixer grinder.

The extraction was carried out by using a magnetic stirrer. 100 gm mushroom powder was mixed with 1 liter Milli Q water and kept on a magnetic stirrer at 60°C for 72 hours. The extract was collected in a separate beaker and filtered twice with Whatman no. 1 filter paper. The liquid extract was dried at 60°C temperature with the help of a water bath and stored at 4°C until used. To prevent any potential harm to the animal's organs, we opted for an aqueous extract. Numerous studies have documented the negative impact of methanol and other organic solvents on liver and kidney function [13, 14], which could compromise the accuracy of our results. Additionally, we chose water as the solvent because it can be easily redissolved in water, unlike other solvent extracts that may not dissolve entirely due to their extraction in alternative solvents.

### 2.2. Animals

Male Wistar rats of 175-200 g of body weight and age of 9 weeks were used in this study. The animals were housed in controlled conditions and were provided 12 : 12 hours of light and dark cycles. The animals were divided into five different experimental groups (normal, diabetic, drug, T1, and T2) as per our previous study [12]. The animals were given standard feed, purchased from New Delhi, India, and water ad libitum.

### 2.3. Experiment Design

During this study, 30 animals were divided into five different experimental groups, in which group I was normal to control and received normal saline, and groups II, III, IV, and V were diabetic control, drug control, T1, and T2, respectively. Where the drug control group received metformin (100 mg/kg of body weight) as a standard drug, T1 and T2 groups were dosing groups that received *P. fossulatus* aqueous extract in 250 mg/kg and 500 mg/kg of body weight concentrations, respectively. The dose was selected based on the literature survey and the availability of the sample [15]. Diabetic experimental groups were developed by giving the dose of 60 mg/kg STZ intraperitoneal (IP) injection. The STZ was freshly prepared in 0.1 M ice-cold citrate buffer. All doses of standard medicine and extract were given orally for 21 days. At the end of the experiment, the animals were sacrificed, and organs and tissue were kept in a 10% formalin solution.

### 2.4. Histoslide Preparation of the Kidney and Liver

The followed methodology was based on the protocol described by Yawu et al. [16] with slight modifications. Kidney and liver were removed from all the groups, which were washed with normal saline and stored in 10% formalin. The mixture of absolute alcohol and xylene in a 1 : 1 ratio was prepared, and organs were placed into it for 20 minutes. Then again, tissues were put into a xylene solution for 30 minutes. The paraffin blocks, containing organs, were prepared, and by using a microtome, 5 *μ*m thickness sections were cut. The sections were transferred onto the glass slides and then dewaxed with the help of a xylene solution. The prepared slides were stained with hematoxylin for 30 seconds, counterstained by using eosin, and then mounted. All the images of the liver and kidney histoslides were taken at 20x and 40x (from Olympus microscope; modal; CKX53, camera model; Megcam-MU2A).

## 3. Results

### 3.1. Effect of *P. fossulatus* on the Kidney

The kidney of the normal control group had normal structures of proximal, distal tubules, and glomerulus which was surrounded by Bowman's capsule (Figure 1). In Figure 2, at 40x, the structures of the glomerulus could be seen clearly. There were no signs of mesangial cell expansion. There was no injury or inflammation observed in proximal convoluted tubules. In the diabetic control group, Figure 1, at 20x, Bowman's space was more compared with the normal control group. The expansion of mesangial cells and tubular atrophy were observed clearly in Figure 2, at 40x resolution, whereas in the drug control group, a few glomeruli were damaged, but the overall structures were improved (Figure 1). The mesangial cell expansion seems to be improved compared with the normal and diabetic control groups. Bowmen's capsule was also found normal (Figure 2). In the test groups, i.e., T1 and T2 groups, glomeruli improved, compared with the normal and diabetic control groups. However, a few glomeruli were found to be damaged, and the rest were recovered and improved (Figures 1 and 2). In the T1 group, tubular atrophy was observed (Figure 2).

### 3.2. Effect of *P. fossulatus* on the Liver

The normal control group showed regular and natural structures of hepatocytes and sinusoids along with the portal triad. The hepatic architecture morphology was also found normal. There were no signs of injury or damage to the organ (Figure 3) which was confirmed in Figure 4, at 40x resolution. In the diabetic control group, the irregular structure of hepatocytes and necrosis were observed in Figure 3, 20x, whereas some other changes like sinusoidal dilatation, more numbers of the Kupffer cells, and monocytes were also observed in Figure 4, at 40x resolution. The drug control group showed no signs of necrosis and improvement in sinusoidal dilatation, and fewer numbers of the Kupffer cells were observed (Figures 3 and 4). Dosing groups, T1 and T2, showed improved architectures of hepatocytes and improvement in sinusoidal dilatation. However, necrosis was observed in the T1 group. The T2 group showed much more improvements in histological changes, and there were no signs of necrosis found (Figures 3 and 4).

## 4. Discussion

DM is one of the most complicated diseases that can cause serious health-related problems, and if it is untreated and uncontrolled, then it may lead to death also. There are more than 390 million people worldwide suffering from diabetes, and it is expected to rise this number to about 500 million people by 2030 [17]. There is no permanent and definite treatment available for DM. Although some therapies are used to manage the adverse effects of DM, these are also causing serious side effects on the organs of the patients. The liver and kidney are the prime targets of DM. These organs showed many histopathological changes. If the diabetes is uncontrolled, then it may lead to ESRD in the kidney, a condition of DN. Due to hyperglycemic conditions, the liver can also be associated with many diseases like cirrhosis and NAFLD.

People are preferring natural and fewer side-effect-causing medicines. The aqueous extract of *P. fossulatus* has shown its potential in reducing the blood glucose level and improving the functions of the kidney and liver in our previous study [12]. However, the biomolecules of *P. fossulatus* are still needed to be identified. The aqueous extract of *P. fossulatus* and its effects on histopathological changes were evaluated in detail in this study.

STZ targets the *β*-cells of the pancreas due to which impaired secretion of insulin occurs, leading to the onset of diabetes mellitus. STZ is used to induce diabetes in rats because it shows some other clinical symptoms like weight loss, polyuria, hyperlipidemia, and hyperphagia [18]. All the above symptoms are the same as can be seen in human patients; maybe this is the reason for using STZ to induce diabetes in animals. In diabetic conditions, animals showed the development of nephropathy, the same as an early stage of nephropathy in humans [19].

The histological changes observed in the kidney histoslides were damage to the glomerulus, which helps in infiltration function, and this function is hampered if the glomerulus is damaged. Due to these reasons, glycogen is deposited in the cells, leading to cell damage. However, *P. fossulatus* aqueous extract helps to protect the glomerulus cells and reduce glycogen deposition. The results of this study have been compared with the results of Teoh et al. [20], where they used the extract of *Momordica charantia* to explore the histological changes in the kidney of diabetic rats and found that the treated group of animals had normal basement membrane with normal glomerulus which is similar to our findings.

During the experiments in the diabetic control group, the Kupffer cells were observed in large numbers which indicate the damage of liver cells which is similar to the findings of the study done by Ahmed et al. [21]. A few numbers of monocytes were also observed, whereas in the drug control and dosing group T2, the monocytes and the Kupffer cells were found in very less numbers. The Kupffer cells are macrophages found in the liver and release chemotoxines and cytotoxins. The Kupffer cells play a very important role against infectious disease, fatty liver disease, liver injury, and liver fibrosis [22]. The Kupffer cells get activated, releasing IL-1 and TNF-*α*, which further activates the expression of endothelial sinusoidal ICAM-1 and leukocytes. This results in damage to the endothelium [23]. Balamash et al. [24] did a study on metformin and virgin olive oil efficacy against STZ-induced diabetic Sprague-Dawley Rats, in which they found the same kind of results, validating the results of our study.

The aqueous extract of *P. fossulatus* protects the kidney and liver which are the vital organs of the body, and due to these attributes, this mushroom has proven to be a good antihyperglycemic agent. However, the exact mechanism needs to be uncovered.

## 5. Conclusion

In conclusion, the aqueous extract showed its efficacy in the protection of the kidney and liver in the STZ-induced diabetic rat model from harmful side effects of diabetes. The extract helps to improve organ functions by recovering its histopathological changes. It restored the structural functions of the kidney and liver to near their natural shape. The possible mechanism of protective effects maybe would induce the damage repair mechanism of the cells so that the cells repair the damaged part. Hence, we can use *P. fossulatus* either with traditional therapy or alone for the management of diabetes. The limitation of the present study is using H&E staining because it does not provide information about the biological molecules and distribution of cytoplasmic chemicals that could be more useful in the visualization of the cell morphology and structures.

## Figures and Tables

**Figure 1:** Kidney histology at 20x resolution. All the groups were stained with H&E (20x) and observed the glomerulus which is the most effective area of the kidney due to diabetes. (a) The normal control group had a regular structure of glomerulus, and (b) the diabetic control group, (c) the drug control group, and (d) the D1 and (e) D2 groups observed irregular shapes. Green arrows show glomerulus structure in different groups.

**Figure 2:** Kidney histology at 40x resolution showed a much more clear picture. All the groups were stained with H&E (40x) and observed at higher magnificence (a) the normal control group had the normal and regular structure of glomerulus, and (b) the diabetic control group, (c) the drug control group, and (d) the D1 and (e) D2 groups were experimental. Green arrows show tubular atrophy; light blue arrows show space between Bowmen's capsule membrane; yellow arrows show mesangial expansion.

**Figure 3:** Liver histology at 20x resolution. All the groups were stained with H&E (20x). All the images were taken in such a way that it covers the major affected area of the liver. The main consideration areas were the portal triad, central vein, and the numbers of the Kupffer cell expression. (a) the normal control group, (b) the diabetic control group, (c) the drug control group, and (d) the D1 and (e) D2 groups. Green arrows show the portal triad; light blue arrows show the central vein; dark brown arrows show necrosis; black arrows show the Kupffer cells.

**Figure 4:** Liver histology at 40x resolution. All the groups were stained with H&E (400x). All the images were taken at a higher resolution so that they showed affected areas much more clearly. (a) the normal control group had normal cell structure, whereas the experimental groups (b) the diabetic control group, (c) the drug control group, and the (d) D1 and (e) D2 groups showed necrosis and major morphological changes. Green arrows show the portal triad; light blue arrows show the central vein; black arrows show the Kupffer cells; dark blue showing sinusoids.

## Data Availability

They can be shared by the corresponding author on valid requests.
